# Effects of Knee Debridement with Flurbiprofen on Knee Function, Inflammatory Levels, and Bone Metabolism Activity in Patients with Knee Osteoarthritis

**DOI:** 10.1155/2022/8031360

**Published:** 2022-07-01

**Authors:** Tao Lin, Zemiao Liu, Wei Ji, Peng Zhang

**Affiliations:** Department of Joint Surgery, Qilu Hospital (Qingdao), Cheeloo College of Medicine, Shandong University, 266035 Qingdao, Shandong Province, China

## Abstract

**Objective:**

The objective of this study is to explore the effects of knee debridement with flurbiprofen on the knee function, inflammatory levels, and bone metabolism activity in patients with knee osteoarthritis.

**Methods:**

110 patients with knee osteoarthritis who underwent arthroscopic debridement in our hospital from 2020.01 to 2022.01 were selected for retrospective analysis. Based on whether or not flurbiprofen was used in combination during the perioperative phase, the patients were divided into the control group (only arthroscopic debridement of the knee) and the research group (flurbiprofen with arthroscopic debridement of the knee), with 55 cases in each group. The indexes such as knee function, inflammatory levels, and bone metabolism activity of the two groups were analyzed.

**Results:**

According to hospital for special surgery (HSS) evaluation for knee function, most patients in the control group were assessed as “moderate,” while patients in the research group were mainly focused on “excellent” and “good,” and their excellent and good rates were remarkably higher than those in the control group (*P* < 0.05). There were no significant variations in bone metabolism indices such as osteoprotegerin levels (OPG), insulin-like growth factor-1 (IGF-1), *β*-isomerized C-terminal telopeptide (*β*-CTX), and receptor activator of nuclear factor-*κ*B ligand (RANKL) before treatment between both groups (*P* > 0.05), with higher OPG, IGF-1 levels, and remarkably lower *β*-CTX, RANKL levels in the research group than those in the control group after treatment (*P* < 0.05). There were no remarkable differences in pain between both groups before treatment (*P* > 0.05), while at 24 h and 48 h after surgery, the VAS scores in the research group were remarkably lower than those in the control group (*P* < 0.05). In terms of inflammatory factors, the levels of interleukin-1*β* (IL-1*β*), tumor necrosis factor-*α* (TNF-*α*), and cyclooxygenase-2 (COX-2) in the research group were remarkably lower than those in the control group after treatment (*P* < 0.05).

**Conclusion:**

Arthroscopy coupled with flurbiprofen provides a good analgesic effect in the therapeutic treatment of patients with knee osteoarthritis, which contributes to the recovery of knee function with definite results. Its mechanism may be associated with the control of inflammatory response and the regulation of bone metabolism disorder.

## 1. Introduction

Knee osteoarthritis is a chronic join disease of the knee where the inflammation progresses slowly, and symptoms such as knee pain, swelling, stiffness, and deformity gradually develop, which affect the daily activities of patients and may render them completely immobile in the worst-case scenario [1–3]. Currently, the treatment of knee osteoarthritis is aimed at relieving pain, delaying disease progression, correcting deformities, improving or restoring joint function, and improving patients' quality of life. In clinical practice, laddering, personalized, and comprehensive treatments are taken as the leading treatment protocols, including four levels of basic, pharmacological, restorative, and reconstructive treatment [4–6]. Basic treatment, which is suitable for all patients with knee osteoarthritis, is only required by very few patients in the early stages with mild symptoms in the form of health education, exercise, and physical therapy. Most patients with clinical diagnosis need to receive pharmacological, restorative, or even reconstructive treatment. Pharmacological treatment includes many types such as external use, oral administration, intravenous infusion, and intraarticular injection, for the main purpose of analgesia and symptom relief. Restorative treatment like arthroscopic debridement can remove many pain-causing factors, control the disease, prolong the use of joints, and avoid premature joint replacement surgery [7–9]. However, knee debridement cannot not cure the disease, and many patients still have obvious joint swelling and pain after surgery. Since knee debridement is performed under local anesthesia, the perioperative analgesic management of such patients is particularly important for the prognosis and has always been a major clinical research challenge. Flurbiprofen is a nonsteroidal anti-inflammatory analgesic drug with certain targeting effects, and several studies have shown its good efficacy on the pain after orthopedic surgery [10, 11]. It can be used for preemptive analgesia or postoperative analgesia, but there are few studies on flurbiprofen-assisted arthroscopic debridement for knee osteoarthritis. This study intends to observe the effects of flurbiprofen on knee function and bone metabolism indexes in patients with knee osteoarthritis during the perioperative period of arthroscopic debridement.

The paper's organization paragraph is as follows: The materials and methods are presented in Section 1.  Section 2, discusses the experiments and results. Finally, in Section 3, the research work is concluded with discussion.

## 2. Materials and Methods

### 2.1. Inclusion and Exclusion Criteria

Inclusion criteria are as follows: ① The patients met the therapeutic indications of knee arthroscopic debridement; ② the patients were aged ≥50; ③ the patients had no contraindications to flurbiprofen; ④ the patients were ranked in class I-II by ASA; ⑤ the patients had no peripheral neuropathy; ⑥ the patients had no history of peptic ulcer; and ⑦ the patients and their family members knew the study protocol and signed the consent form.

Exclusion criteria are as follows: ① patients with abnormal coagulation function; ② patients with cardiac or renal insufficiency; ③ patients with immune or infectious diseases; ④ patients with cognitive impairment or psychiatric diseases; ⑤ patients who dropped out after surgery; ⑥ patients with a history of allergy to nonsteroidal anti-inflammatory drugs; and ⑦ patients with long-term preoperative use of other analgesic drugs.

### 2.2. Selection and Grouping of Patients

The research objects were selected from the patients with knee osteoarthritis who underwent arthroscopic debridement in our hospital from 2020.01 to 2022.01, with the total sample size of 110 cases. The patients were grouped according to whether flurbiprofen was used in combination during the perioperative period. In other words, the patients who underwent arthroscopic debridement of the knee only were placed in the control group, and those who also received flurbiprofen treatment were placed in the research group, with 55 cases in each group. The study conformed to the ethical and moral standards of our hospital and was approved by the Ethics Committee.

### 2.3. Method

#### 2.3.1. Arthroscopic Debridement

Continuous epidural anesthesia or subarachnoid block anesthesia was administered, and balloon tourniquets (37.2-43.9 kPa) were used. The approaches for knee followed Jackson' s standard. Arthroscope and surgical instruments were placed medially and laterally under the patella, and 1 L of 0.1% epinephrine injection and 3000 ml of normal saline were perfused through the suprapatellar lateral incision. The intraarticular conditions were explored under an arthroscope, with several treatments as follows: ① Treatment of cartilage injury. Cartilage injury was graded by Outerbridge scale. Injury of grade 1 was not treated specially; injury of grades 2-3 was trimmed with a cartilage shaver and treated with radiofrequency and gasification; grade 4 injuries were treated with a curette or nucleus pulposus clamp to remove the unstable cartilage edge, followed by radiofrequency, gasification, and solidification. ② Treatment of lateral patellar retinaculum. The patients who had obvious patellar subluxation or lateral tilt, and reduced mobility with obvious tenderness over lateral retinaculum by preoperative axial X-ray, and had degeneration of the lateral cartilage with intact medial cartilage according to arthroscopy, were treated with lateral retinacular release. ③ Treatment of osteophytes. Osteophytes that blocked flexion and extension of joints and caused frictional damage on articular cartilage surface were removed by grinding. ④ Treatment of hyperplastic synovium. Severely congested and edematous synovium, significantly thickened infrapatellar fat pad, and fat pad or synovium that affected joint flexion and extension and had obvious tenderness before surgery were moderately shaved and resected. ⑤ Treatment of meniscus injury. Partial or subtotal resection was conducted in the patients who had degenerative meniscus tears, trying to retain the anterior horn and removing the free body and debris. After cleaning, the joint cavity was repeatedly flushed with plenty of normal saline, and the knee joint was bandaged. All patients received arthroscopic debridement of the knee by the same group of physicians.

#### 2.3.2. Flurbiprofen

50 mg of flurbiprofen was intravenously injected before surgery (specification. 5 ml: 50 mg, Beijing Tide Pharmaceutical Co., Ltd., NMPA Approval No. H20041508) for analgesia. For 24-h postoperative continuous analgesia, the analgesic pumps were given 100 mL of 0.2% ropivacaine, and flurbiprofen was injected intravenously once every 12 h, with 50 mg each time.

### 2.4. Observation Indexes

#### 2.4.1. General Data

Age, BMI, gender, affected side, underlying diseases (diabetes, hypertension, and hyperlipidemia), ASA classification, and K-L classification were the main statistical data.

#### 2.4.2. Knee Function

After treatment, the patients' knee function was evaluated according to the hospital for special surgery (HSS) scoring system, where the six evaluation dimensions included pain (30 points), function (22 points), range of motion (18 points), muscle strength (10 points), knee flexion deformity (10 points), and knee instability (10 points). Knee function was graded and scored by the clinical efficacy, with 85 points or more as excellent; 70-84 as good; 60-69 as moderate; and below 59 as poor.

3 ml fasting venous blood of the patients was taken in the early morning. The levels of interleukin-1*β* (IL-1*β*), tumor necrosis factor-*α* (TNF-*α*), cyclooxygenase-2 (COX-2), insulin-like growth factor-1 (IGF-1), osteoprotegerin (OPG), and receptor activator of nuclear factor-*κ*B ligand (RANKL) were detected based on enzyme-linked immunosorbent assay. The level of *β*-isomerized C-terminal telopeptide (*β*-CTX) was detected by electrochemiluminescence immunoassay.

#### 2.4.3. Pain

The patients' degree of pain was evaluated by visual analog scale (VAS) which uses a 10-cm-long straight line or ruler with 0 reflecting “no pain” and 10 reflecting the “worst pain” at either end. The patients marked the numbers on the straight line according to the pain they felt to indicate the intensity of pain and the degree of psychological displeasure, with 0 as no pain, 1-3 as mild pain, 4-6 as moderate pain, 7-9 as severe pain, and 10 as intolerable pain, i.e., severe pain.

### 2.5. Statistical Disposal

In this study, the differences between both groups were calculated by SPSS20.0, with the images edited based on GraphPad Prism 7 (GraphPad Software, San Diego, USA). The research data consisted of count data and measurement data, which were expressed as [*n* (%)] and (^−^*x* ± *s*) and tested by *X*^2^ and *t* tests. The differences were statistically remarkable when *P* < 0.05.

## 3. Results

### 3.1. General Data

There is no remarkable difference in the data such as mean age, BMI, gender, affected side, underlying diseases (diabetes, hypertension, hyperlipidemia), ASA classification, and K-L classification between both groups (*P* > 0.05), which was detailed in Table 1.

### 3.2. Knee Function

According to the HSS evaluation for knee function, most patients in the control group are assessed as “moderate,” while patients in the research group are mainly focused on “excellent” and “good,” and their excellent and good rates are remarkably higher than those in the control group (*P* < 0.05), which is detailed in Table 2.

### 3.3. Bone Metabolism

There is no remarkable difference in the levels of bone metabolism indexes such as OPG, IGF-1, *β*-CTX, and RANKL between both groups before treatment (*P* > 0.05), with higher OPG, IGF-1 levels, and remarkably lower *β*-CTX, RANKL levels in the research group than those in the control group after treatment (*P* < 0.05), which is detailed in Table 3.

### 3.4. Pain

There are no remarkable differences in pain between both groups before treatment (*P* > 0.05), while at 24 h and 48 h after surgery, the VAS scores in the research group are remarkably lower than those in the control group (*P* < 0.05), which is detailed in Figure 1.

### 3.5. Inflammatory Factor Levels

In terms of inflammatory factors, the levels of IL-1*β*, TNF-*α*, and COX-2 in the research group are remarkably lower than those in the control group after treatment (*P* < 0.05), with statistically remarkable differences, which is shown in Table 4.

## 4. Discussion

Arthroscopic debridement has the advantages of minimal invasion, rapid postoperative recovery, and low cost, making it one of the common treatments for knee osteoarthritis. But the invasive nature of arthroscopic debridement inevitably leads to the intraoperative damage of intraarticular tissues which induces local swelling, adhesions, and inflammatory reactions. Furthermore, arthroscopic debridement, which is frequently accompanied with medicines for total treatment in clinic, is often challenging for patients with severe knee osteoarthritis to achieve excellent results [12–14]. In addition, perioperative analgesia for such patients is also an important way to alleviate postoperative pain and guarantee that the early postoperative functional exercise goes through smoothly. According to relevant reports, most patients with knee osteoarthritis show obvious local inflammatory injury and severe postoperative pain after arthroscopic debridement, which is attributed to intraoperative tissue damage and inflammatory response. Flurbiprofen is a nonselective, nonsteroidal anti-inflammatory drug that targets injury sites of tissues and vessels, selectively reduces the level of inflammatory factors in the blood circulation, and has certain targeted anti-inflammatory and analgesia effects which have been demonstrated in several postoperative analgesia studies [15–17]. In this study, patients with knee osteoarthritis in our hospital were chosen as the subjects for research, in order to further explore the effects of arthroscopic debridement with flurbiprofen on keen function and bone metabolism indexes and its mechanism.

During the perioperative period of arthroscopic debridement, the patients in the research group were given flurbiprofen. There were no remarkable differences in pain between both groups before treatment (*P* > 0.05), while at 24 h and 48 h after surgery, the VAS scores in the research group were remarkably lower than those in the control group (*P* < 0.05), which was consistent with the report of Nichilas Bene et al. [18]. As a nonsteroidal anti-inflammatory analgesic, flurbiprofen can reduce prostaglandin production by inhibiting central and peripheral cyclooxygenase, achieving analgesic effects, and reducing nociceptive sensitivity caused by surgical stimulation, as well as suppressing the release of inflammatory factors. Subsequently, this study found that the levels of inflammatory factors such as IL-1*β*, TNF-*α*, and COX-2 were remarkably lower in the research group than in the control group after treatment (*P* < 0.05). The occurrence of knee osteoarthritis is mainly related to degenerative joint lesions or metabolic disorders, while inflammatory factors also play an important role in it. TNF-*α* is a pro-inflammatory cytokine that can increase osteoclast activity and inhibit osteoblast activity, inhibit the synthesis of proteoglycans and cartilage collagen, and is involved in the occurrence and development of knee osteoarthritis. IL-1*β* is a hormone-like peptide inflammatory factor, which also participates in the process of cartilage apoptosis. COX-2 is a rate-limiting enzyme synthesized by prostaglandins, which is highly expressed under the induction of IL-1, TNF-*α*, or other cytokines. Some studies have found that the high expression of COX-2 in local joint is an important factor leading to knee osteoarthritis, whose progression is also accompanied by the further increased expression level of COX-2 [19–21]. As a result, the findings suggest that combining flurbiprofen perioperatively with arthroscopic debridement in individuals with knee osteoarthritis is helpful, especially for reducing the expression of IL-1*β*, TNF-*α*, COX-2, and other inflammatory factors. In addition, the imbalance of bone metabolism is also an important aspect reflecting local bone destruction and systemic bone loss in patients with osteoarthritis. Osteogenesis-osteolysis imbalance is mainly manifested as bone reconstruction, abnormal activation of osteoclasts, and imbalance of bone resorption and bone formation, and thus, the levels of OPG, IGF-1, *β*-CTX, RANKL, and other bone metabolism indexes in peripheral serum will change abnormally. This study found that the levels of OPG and IGF-1 were higher (*P* < 0.05), and the levels of *β*-CTX and RANKL were remarkably lower (*P* < 0.05) in the research group than in the control group after treatment. *β*-CTX is a bone resorption marker and shows a remarkable positive correlation with the degree of joint pain and swelling in patients. IGF-1 can reflect the activity of osteoblasts and has a significant role in the repair of damaged cartilage. OPG can block the binding of RANKL to RANK, inhibit osteoclast differentiation and maturation, and thus inhibit bone resorption [22–25]. The findings show that flurbiprofen combined with arthroscopic debridement is more effective in managing bone metabolism abnormalities and enhancing knee function recovery in patients with knee osteoarthritis. Then, according to the HSS evaluation for knee function, it was found that most patients in the control group were assessed as “moderate,” while patients in the research group were mainly focused on “excellent” and “good,” and their excellent and good rates were remarkably higher than those in the control group (*P* < 0.05). It suggested that flurbiprofen combined with arthroscopic debridement is effective in patients with knee osteoarthritis and has a greater potential application for their prognostic recovery.

To sum up, for patients with knee osteoarthritis, flurbiprofen combined with arthroscopic debridement is effective and has good analgesic effect, which contributes to the recovery of knee function. Its mechanism may be associated with the control of inflammatory reaction and the regulation of bone metabolism disorder.

## Figures and Tables

**Figure 1:** Results of VAS scores. Notes: The transverse axis was time points, and the longitudinal axis was the VAS score (points). The VAS scores in the control group before surgery, 24 h after surgery, and 48 h after surgery were (6.07 ± 1.09) points, (4.82 ± 0.81) points, and (3.73 ± 1.02) points, respectively. The VAS scores in the research group before surgery, 24 h after surgery, and 48 h after surgery were (6.07 ± 1.04) points, (2.95 ± 0.62) points, and (1.87 ± 0.74) points, respectively. ∗ suggested remarkable differences in the VAS scores at 24 h after surgery between both groups (*t* = 13.596, *P* < 0.001). ∗∗ suggested remarkable differences in the VAS scores at 48 h after surgery between both groups (*t* = 10.946, *P* < 0.001).

**Table 1:** Comparison of general data (*n* = 55).

Observation indexes	Control group	Research group	*X* ^2^/*t*	*P*
Age (years)	62.20 ± 4.70	61.95 ± 4.57	0.283	0.778
BMI (kg/m^2^)	23.15 ± 3.01	23.26 ± 3.04	0.191	0.849
Gender			0.334	0.563
Male	25 (45.54)	22 (40.00)		
Female	30 (54.55)	33 (60.00)		
Affected side				
Left side	21 (38.18)	17 (30.91)	0.643	0.423
Right side	27 (49.09)	30 (54.55)	0.328	0.567
Both sides	7 (12.73)	8 (14.55)	0.077	0.781
Underlying diseases				
Diabetes	27 (49.09)	25 (45.45)	0.146	0.702
Hypertension	29 (52.73)	30 (54.55)	0.037	0.848
Hyperlipidemia	24 (43.64)	23 (41.82)	0.037	0.847
ASA classification			0.334	0.563
Class I	22 (40.00)	25 (45.45)		
Class II	33 (60.00)	30 (54.55)		
K-L classification				
Class II	24 (43.64)	26 (47.27)	0.147	0.702
Class III	25 (45.45)	24 (43.64)	0.037	0.848
Class IV	6 (10.91)	5 (9.09)	0.101	0.751

**Table 2:** Results of HSS evaluation.

Groups	Excellent	Good	Moderate	Poor	Excellent and good rate
Control group	8 (14.55)	11 (20.00)	25 (45.45)	11 (20.00)	19 (34.55)
Research group	19 (34.55)	22 (40.00)	10 (18.18)	4 (7.27)	41 (74.55)
*X* ^2^					17.747
*P*					<0.001

**Table 3:** Results of bone metabolism indexes.

Indexes	Control group	Research group	*t*	*P*
OPG (pg/ml)				
Before treatment	3.12 ± 0.71	3.16 ± 0.82	0.273	0.785
After treatment	4.63 ± 0.72	5.41 ± 0.66	5.922	<0.001
IGF-1 (*μ*g/L)				
Before treatment	75.56 ± 6.32	75.82 ± 6.50	0.213	0.832
After treatment	86.25 ± 7.91	92.03 ± 8.01	3.808	<0.001
*β*-CTX (pg/ml)				
Before treatment	0.92 ± 0.25	0.93 ± 0.24	0.214	0.831
After treatment	0.75 ± 0.21	0.45 ± 0.12	9.199	<0.001
RANKL (pg/ml)				
Before treatment	48.75 ± 4.15	48.62 ± 4.08	0.166	0.869
After treatment	38.56 ± 3.15	30.01 ± 2.43	15.938	<0.001

**Table 4:** Results of inflammatory factor levels.

Groups	Cases	IL-1*β* (ng/L)	TNF-*α* (pg/ml)	COX-2 (pg/ml)
Control group	55	4.79 ± 1.07	7.02 ± 1.28	16.65 ± 2.34
Research group	55	3.72 ± 1.05	5.47 ± 1.19	12.43 ± 2.10
*t*		5.293	6.577	9.954
*P*		<0.001	<0.001	<0.001

## Data Availability

Data to support the findings of this study is available on reasonable request from the corresponding author.

## References

[1] Yiallourides C., Naylor P. A. (2021). Time-frequency analysis and parameterisation of knee sounds for non-invasive detection of osteoarthritis. *IEEE Transactions on Biomedical Engineering*.

[2] Nguyen C., Rannou F. (2017). The safety of intra-articular injections for the treatment of knee osteoarthritis: a critical narrative review. *Expert Opinion on Drug Safety*.

[3] Boonhong J., Suntornpiyapan P., Piriyajarukul A. (2018). Ultrasound combined transcutaneous electrical nerve stimulation (UltraTENS) versus phonophoresis of piroxicam (PhP) in symptomatic knee osteoarthritis: a randomized double-blind, controlled trial. *Journal of Back and Musculoskeletal Rehabilitation*.

[4] Mukhopadhyay K., Ghosh P., Ghorai P., Hazra A., Das A. K. (2018). Oxaceprol versus tramadol for knee osteoarthritis: a randomized controlled trial. *Indian Journal of Pharmacology.*.

[5] Singh S., Pattnaik M., Mohanty P., Ganesh G. S. (2016). Effectiveness of hip abductor strengthening on health status, strength, endurance and six minute walk test in participants with medial compartment symptomatic knee osteoarthritis. *Journal of Back and Musculoskeletal Rehabilitation*.

[6] Kim S. H., Cho W.-S., Joung H.-Y., Choi Y. E., Jung M. (2017). Perfusion of the rotator cuff tendon according to the repair configuration using an indocyanine green fluorescence arthroscope: a preliminary report. *American Journal of Sports Medicine*.

[7] Kim N., Jung S. B. (2019). Percutaneous unilateral biportal endoscopic spine surgery using a 30-degree arthroscope in patients with severe lumbar spinal stenosis-a technical note. *Clinical Spine Surgery*.

[8] Kwon B. C., Lee J.-K., Lee S. Y., Hwang J. Y. (2019). Does use of the 70° arthroscope improve the outcomes of arthroscopic debridement for chronic recalcitrant tennis elbow?. *Journal of Shoulder and Elbow Surgery*.

[9] Wahl E. P., Coughlin R. P., Mickelson D. T., Green C. L., Garrigues G. E. (2019). How arthroscope orientation affects performance. *The Journal of Bone and Joint Surgery. American Volume*.

[10] Mariani P. P. (2019). The 45 degrees arthroscope: a forgotten scope in knee surgery. *Revue de Chirurgie Orthopédique et Traumatologique*.

[11] Maffulli N. (2018). *Editorial commentary:* hip trochanteric bursitis and femoroacetabular impingement: the arthroscope is only the tool. *Arthroscopy*.

[12] Dahmen J., Kerkhoffs G. M. M. J., van Bergen C. J. A. (2021). *Editorial commentary*: how far can the arthroscope reach in the ankle joint?. *Arthroscopy: The Journal of Arthroscopic and Related Surgery*.

[13] Koc B., Somorjai N., Kiesouw E. P. (2017). Endoscopic debridement and fibrin glue injection of a chronic Morel-Lavallee lesion of the knee in a professional soccer player: a case report and literature review. *The Knee*.

[14] Ottesen C. S., Troelsen A., Sandholdt H., Jacobsen S., Husted H., Gromov K. (2019). Acceptable success rate in patients with periprosthetic knee joint infection treated with debridement, antibiotics, and implant retention. *The Journal of Arthroplasty*.

[15] Vahedi H., Aali-Rezaie A., Shahi A., Conway J. D. (2019). Irrigation, debridement, and implant retention for recurrence of periprosthetic joint infection following two-stage revision total knee arthroplasty: a matched cohort study. *The Journal of Arthroplasty*.

[16] Duque A. F., Post Z. D., Lutz R. W., Orozco F. R., Pulido S. H., Ong A. C. (2017). Is there still a role for irrigation and debridement with liner exchange in acute periprosthetic total knee infection?. *The Journal of Arthroplasty*.

[17] Jourdan M. (2018). Risk factors for repeat debridement, spacer retention, amputation, arthrodesis, and mortality after removal of an infected total knee arthroplasty with spacer placement. *The Journal of Arthroplasty*.

[18] Bene N., Li X., Nandi S. (2018). Factors affecting failure of irrigation and debridement with liner exchange in total knee arthroplasty infection. *The Knee*.

[19] Urish K. L., Bullock A. G., Kreger A. M. (2018). A multicenter study of irrigation and debridement in total knee arthroplasty periprosthetic joint infection: treatment failure is high. *The Journal of Arthroplasty*.

[20] Manrique J., Komnos G. A., Tan T. L., Sedgh S., Shohat N., Parvizi J. (2019). Outcomes of superficial and deep irrigation and debridement in total hip and knee arthroplasty. *The Journal of Arthroplasty*.

[21] Paliwal S., Tilak A., Sharma J. (2019). Flurbiprofen-loaded ethanolic liposome particles for biomedical applications. *Journal of Microbiological Methods*.

[22] Isiklan N., Erol U. H. (2020). Design and evaluation of temperature-responsive chitosan/hydroxypropyl cellulose blend nanospheres for sustainable flurbiprofen release. *International Journal of Biological Macromolecules: Structure, Function and Interactions*.

[23] Pande S., Vashi J., Solanki A. (2020). Formulation and characterization of ileo-colonic targeted mucoadhesive microspheres containing flurbiprofen for treatment of ulcerative colitis. *Research Journal of Pharmacy and Technology*.

[24] Alokour M., Yilmaz E. (2021). A polymer hybrid film based on poly(vinyl cinnamate) and poly(2-hydroxy ethyl methacrylate) for controlled flurbiprofen release. *Journal of Polymer Research*.

[25] Oktay A. N., Karakucuk A., Ilbasmis-Tamer S., Celebi N. (2018). Dermal flurbiprofen nanosuspensions: optimization with design of experiment approach and *in vitro* evaluation. *European Journal of Pharmaceutical Sciences*.

